# Influence of COVID-19 on the Tourism Industry in China: An Artificial Neural Networks Approach

**DOI:** 10.1155/2022/9581387

**Published:** 2022-04-08

**Authors:** Waleed, Zongguo Ma, Fazli Wahid, Samad Baseer, Ahmad Ali AlZubi, Hizbullah Khattak

**Affiliations:** ^1^Business School, Shandong Normal University, Shandong, China; ^2^Department of Information Technology, University of Haripur, Haripur 22620, Khyber Pakhtunkhwa, Pakistan; ^3^Department of Computer System Engineering, University of Engineering and Technology, Peshawar 25000, Pakistan; ^4^Computer Science Department, Community College King Saud University, P.O. Box 28095, Riyadh 11437, Saudi Arabia; ^5^Department of Information Technology, Hazara University Mansehra, Mansehra 21120, Khyber Pakhtunkhwa, Pakistan

## Abstract

Prior to COVID-19, the tourism industry was one of the important sectors of the world economy. This study intends to measure the perception of Chinese tourists concerning the spread of COVID-19 in China. The crowding perception, xenophobia, and ethnocentrism are the measurement indicators of the study. A five-point Likert scale is used to predict the perception of the tourists in various destinations. The Kaiser–Mayer–Olkin test and Cronbach's alpha are conducted to ensure the validity and reliability of the corresponding items. SPSS version 21 is used to obtain factor loading, mean values, and standard deviation. Regression analysis is used to measure the strength of the constructs' relationship and prove the hypotheses. Questionnaires have been filled from 730 Chinese respondents. Artificial neural networks and confusion matrices are used for validation and performance evaluation, respectively. Results show that crowding perception, xenophobia, and ethnocentrism caused the spread of COVID-19 during the epidemic. Hence, the tourism industry in China is adversely affected by COVID-19. The crisis management stakeholders of the country need to adopt policies to reduce the spread of COVID-19. The tourism sector needs to provide confidence to the tourists. It will provide ground for the mental strength of the tourists in China.

## 1. Introduction

COVID-19 has negatively influenced the tourism sector all over the world, causing the shutdown of a large number of tourism destinations [1, 2]. The tourism industry is considered to be the most vulnerable industry to the pandemic. Therefore, a huge effort has been done to reopen the industry but it is not done because of the spreading of the disease [1, 3]. Calamities in the tourism industry are occurring on regular basis [1, 3]. Restricting the spread of pandemics due to COVID-19 has been impossible because of the decline in the tourism and hospitality industry, the collapse of the world economy, variations in tourism sectors, and the predictability of the near future of the tourism industry [4].

In January 2020, COVID-19 got familiar all over the world. The increasing number of confirmed cases made the Chinese government respond quickly to the situation. The whole world was shocked due to the complete lockdown of Wuhan city on January 23, 2020. After one week, the WHO declared the epidemic a public health emergency of international concern (PHEIC) in China. Till that time, the total confirmed cases were 7711, with only 83 cases outside China. China, South Korea, and Iran were the victims of COVID-19. In one week, the cases in South Korea raised from 31 to 1000.

Similarly, the cases in Iran went from zero to 1000 in twelve days. In March, China and South Korea obtained control over the epidemic. In the meantime, it moved to Europe and the United States. The United States had the greatest number of cases, and Italy was with highest fatality rate. The John Hopkins Coronavirus Resource Center data is used to plot the confirmed cases of the six major victim countries. When the WHO announced the pandemic globally, the financial markets were adversely affected. A fall of 30% was observed from February 19 to March 23 in S&P 500. SARS only influenced China, while COVOD-19 has become a crisis for the whole world, showing a more severe impact to be forecasted [5].

Just like the black swan event [6] and World War Two [7], COVID-19 has a significant effect on the global healthcare systems with a waving effect on every aspect of humanity. World Health Organization declared a global emergency on January 30 due to COVID-19 [8]. To overcome the situation, governments have imposed border shutdowns, traveling cancellation, and quarantine [9] in developed countries, fearing the adverse outcomes of economic losses. Because of the economic disorders, primary sectors including industries involved in extracting raw materials, secondary sectors involving finished goods, and tertiary sectors involving services industries have been badly affected [10].

Travelling is considered the most entertaining method of exploring new places in the absence of diseases, criminality, and disasters. Epidemics and pandemics are the two-fearing news for tourists. In such a situation, it is annoying to cope with the situation. Passengers play a vital role in spreading diseases between places [11]. Recently, the world faced an emergency due to the spread of coronavirus. In recent months, the world has been focused on epidemics due to the emergence of a new coronavirus. This virus is highly dangerous and spreads quickly, causing outbreaks all over the world. This virus is transmitted from animals to humans. Severe acute respiratory syndrome (SARS) was transmitted from birds to humans in 2002. The Middle East Respiratory Syndrome (MERS) was transmitted from camels to humans in 2012 [12]. Between November 2002 and June 2003, 8000 people got infected with the SARS virus; two-thirds were from China [13]. Taiwan, Hong Kong, Singapore, and Canada were also affected. Therefore, the tourist avoided visiting Southeast Asia to reduce the risk of infection.

The global value chains have been interrupted because of the production losses in China. Also, China plays an important role in tourism. Chinese tourists spent $277 billion overseas in 2018, 21% of the global spending on tourism [14]. Due to COVID-19, the tourism sector in China has been affected internationally. The lockdown affected the revenue from tourism grippingly. In Thailand, the contribution to GDP in 2018 from tourism was 11%, which was 6% ten years ago. Risk communication works as a good starting point for evaluating expressive forecasts in the tourism sector. Risk communication can explain, educate, and warn about the latent hazards because of information sharing social groups, the information spreading process, or the danger of perceived influence. It also needs to be considered that the quality of information dissemination has a significant impact on risk acceptance and assessments concerning the possibility of occurrence [15].

The most affected industry is hospitality and travel. Marriot International has sent thousands of employees on leave. On March 5, 2020, Hilton Worldwide also informed the creditors to provide $1.75 billion in a revolving loan to overcome financial hardships [16]. The hotel industry revenue per room in the United States fell by 11.6% till March 7, while in China, the occupancy rate reduced by 89% by the end of January 2020. Due to a fall in demand, U.S. hotel companies have planned to provide $150 billion to the staff members in direct assistance and $1.5 billion till February 15 [17]. MGM Resorts International abandoned all kinds of work in Las Vegas on March 16 [18]. The occupancy rates of hotels in Germany declined by 36% since March 1, 2020. The occupancy rate in Italy is also reduced to 6%. London is considered to be the most stable, having an occupancy rate of 47%. Generally, COVID-19 has disturbed the hotel industry significantly [19].

## 2. Literature

Due to the severe conditions of COVID-19, the tourism sector is also affected badly because of the decreasing impacts of supply and demand. The World Travel and Tourism Council has notified that 50 million occupations in the world travel and tourism sector are open to threat [20]. Globally, 1.45 million Chinese visited in the first three months of 2019 to Vietnam, while in January 2020, this figure dropped to 644,000. COVID-19 has brought an evolution in the tourism sector based on epistemology. The central epistemology paradigm in psychology demonstrates human behavior by illuminating its adaptive function and basic intention. As Mayr [21] and Tinbergen [22] explained, evolutionary epistemology differentiates proximate and ultimate motives of human behavior. This approach is termed causation in the field of philosophy [23]. Till now, devastating studies in tourism have focused on proximate approaches to explain human behavior, in that way, ignoring ultimate approaches [24].

Evolutionary psychology claims that humans have inherited physiological and psychological measures apparent in different motives like safety, avoidance from diseases, associations, positions, friend's attainment, friend retaining, and family care [25]. As an explanation of this approach, here, we focus on the avoidance of the coronavirus pandemic. It is vital in tourism research to explain human behavior as a starting opinion for evolution. For instance, a link between the initiation of reproducing approach and a fondness for dangerous traveling activities in humans proposes that risk-taking increases mating accomplishment [26]. Additionally, approaches beyond those explained by Griskevicius and Kenrick [25] exist and play an important part in the behavior of the tourists [24], aimed at an overview of the approach in the tourism research. Tourism is a contemporary activity that is quite different from traditional sociological measures of enhancements and psychological measures that administer the presence of tourism as a pleasant fact [27]. Hence, the researchers aware of latent psychology can ingeniously adopt approaches to tourism based on contemporary measures.

Previous literature shows the value of tourists' capabilities to avoid diseases and perceived health vulnerability related to tourism consequences [28]; Lepp and Gibson, 2003; Reisinger and Mavondo, 2005. These studies are accompanied by insufficient research to examine tourists' assessment and avoidance of infections [29, 30]. Another study investigates the economic and behavioral influence of epidemics and pandemics on tourists [31]; Yang, Zhang, and Chen, 2020; Zhang, Hou, and Li, 2020. Fenichel, Kuminoff, and Chowell (2013) studied that tourists adopted self-protective behavior during the spread of the swine flu epidemic in 2009 and pragmatically related experiences such as apparent vulnerability to avoid traveling [32]. These findings show the significance of avoidance from diseases to understand human behavior on a considerable level.

There exists a connection between disease avoidance, xenophobia, preference for vaccination, and intention for eating local food [33]. Furthermore, the evolutionary tourism paradigm is applicable for providing eventual-level perception for the tourists during the COVID-19 pandemic. Hence, the connection between pandemic and consequences like ethnocentrism, xenophobia, and crowding perceptions is investigated in the tourism literature [34]. As for as COVID-19 is concerned, the island model is applicable because it is an ecological indicator that has abruptly changed the whole world. This concept focuses on the microorganism diseases that are risky for the global environment [35]; Sng et al., 2018. The tourists' behavior has significantly changed due to phenotypic plasticity and ecological variations due to microorganisms. The previous literature has observed a connection between the spread of diseases and tourists' behavior [36].

Both the individual and group level behavioral immune systems have concerns for cognition, affection, and behaviors. An increased prejudice is observed for people with physical disabilities, overweight individuals, and aged people because of unusual characteristics caused by viral diseases [37]. Nevertheless, the human behavioral system is not just affected by others' presence but is also connected with augmented apprehension caused by the potential humiliation [38]. Moreover, the human behavioral immune system has consequences for individuals' behaviors and standards regarding extraversion, sexuality, and candidness to experience [39]. Likewise, microorganisms risk has been connected to enlarged orthodoxy, political traditions, strong family relationships, and religion [40, 41]; Murray and Schaller, 2012. In the case of the behavioral immune system, viral disease catching is more costly than the avoidance to overcome the risk of getting infected [42].

In the previous literature, it has been observed that attitude for gathering fluctuates for individuals. The relationship approach has been connected for preferred marketing areas as a pattern of getting nearer to other people [43]. On the other hand, the initiation of the behavioral immune system enhances the negative perception of the individuals for crowding [30]. The last explanation demonstrates an emerging method for overcoming the influence of the diseases in the crowding areas [30]. Of course, the interpretation of crowded surroundings is applicable to measure revulsion understanding [44]. The literature investigates the perception of the tourists for crowding and experiences [45]; Li, Zhang, Nian, and Zhang, 2017.

Currently, globalization takes place all over the world; xenophobia is harmful because of the avoidance of contact with foreigners but performs certain positive outcomes [37]. Explicitly, xenophobia works to avoid diseases from foreigners to the local people who do not have immunity [46]. Several empirical studies concerning the connection between the behavioral immune system and xenophobia resulted in negative perceptions for foreigners being developed because of the perceived susceptibility to diseases [46, 47]; Prati and Pietrantoni, 2016. Expectedly, such outcomes for xenophobia are predominantly related to major diseases like the Ebola outbreak, which caused vulnerability to the higher American respondents in 2014 [47].

Artificial intelligence (AI) focuses on action, response, or behavior [48]. AI is demonstrated in anthropological and nonanthropological practices to solve problems using learning, analysis, and interpretation of data [49]. AI has developed promptly from doing simple actions to more complex social activities like customers' perception for sustainable intervention [50]. AI is significantly beneficial in reasoning, elaborating, modeling, predicting, and forecasting purposes. As an information technology tool, it is embedded in facilitating customers' internal and external business activities for both personal and impersonal measures [50]. AI is utilized in personal recruitment by combining face recognition and language processing in interviews, training, and development using robots and visual scanning technologies, and salary evaluation using neural networks (Jia et al., 2018). Amazon and Netflix also use AI to analyze customer data and customize products [51].

AI has extensive usage in organizations and industries for bringing evolutionary changes in IT-related fields [50]. For the last ten years, extensive research has investigated technological acceptance and user's satisfaction [52]; King and He, 2006; Marangunić and Granić, 2015; Wixom and Todd, 2005; Wu and Chen, 2017. Practically AI is applicable in customer services to involve customers and develop services in terms of convenience and flexibility. Industrialists and IT advisers are the most important individuals to enhance and apply the role of AI in customer-oriented businesses [51, 53]; Walchuk, 2019. From an IT viewpoint, machines apply AI through learning and natural language processing [54]. From a business perspective, AI administers technologically powered techniques to facilitate business activities for profit maximization [50]. From a user point of view, AI is a collection of instruments for improving efficiency and adding convenience and flexibility to the customers [55]. This study focuses on AI instruments like traveler enhancers and robots in the destinations to provide computer-related services and benefit all the parties, including customers and organizations (de Kervenoael et al., 2020). These instruments are referred to as AI in this study.

AI suggests customer services and provides customer engagement. Affordance theory suggests that AI tools can be applied beneficially in organizations without understanding technological groundwork (Jones, 2003). This theory is originated from ecological research; it can also be applied in organizations to know how technologies can be made realistic in organizations in terms of efficiency, satisfaction, and involvement [56]; Ganguli and Roy, 2011. AI is used to measure that customer response reflects their behavior like satisfaction, purchasing habits, and loyalty. Ajzen (1985) suggested the theory of planned behavior to associate beliefs, attitudes, and behavior in psychology, marketing, and information technology [50, 57, 58]. The current study focuses on applying AI to customer responses rather than behavioral outcomes in the tourism industry. Chatbots can be used in heritage tourism to administer the need and wants of the tourists. Chatbots sometimes involve the customers by providing positive and consistent interaction [51].

Considering the above discussion, it is concluded that tourists' immune system has a strong relationship with the COVID-19 epidemic. Based on the previous literature, it is examined that the behavioral immune system is open to the perceived infection of COVID-19 [47, 59].

## 3. Problem Statement

Due to social distancing, the period of COVID-19 has been considered to be a time of stress and depression for the tourism sector in China. Using artificial neural networks and statistical tools, this study intends to measure the observed response of Chinese tourists during the pandemic. Chinese people perceived that the spread of COVID-19 is caused by crowding, xenophobia, and ethnocentrism in the country. The spread of diseases in the destinations is caused by crowding. Xenophobia produces tourists' perceptions of discomfort and nervousness related to foreigners at the destinations. Similarly, the Chinese have phenomenal norms and values for tourism development in the country. Tourists perceive that they will get an infection of the disease if they visit the destinations. AI is significantly beneficial in reasoning, elaborating, modeling, predicting, and forecasting purposes in the tourism sector. Similarly, the Likert scale is used to measure the satisfaction level of the tourists. Therefore, the artificial neural network is used to measure the perception of Chinese tourists during COVID-19 in connection with statistical analysis.

## 4. Research Methodology

### 4.1. Stages of the Proposed Model

For measuring H1, H2, and H3, data have been acquired from the respondents using questionnaires. As all the data are not valid for ANN and statistical analysis, the acquired data from the tourists *T*_1_,…, *T*_2_,…, *T*_823_ have been preprocessed to get normalization. For getting valid data, the selection, cleaning, removal of the outliers, and removal of missing values have been performed for the data. Then, the consistency of the data for the questionnaire is obtained using Cronbach's alpha. After measuring the consistency, the confirmatory factor analysis, correlation, and regression analysis have been done.

*T*_1_, *T*_2_,…, *T*_n_ are tourists in China, respectively, as shown in Figure 1. H1, H2, and H3 are the hypotheses of the study. CFA is the confirmatory factor analysis.

H1. Crowding influences the spread of COVID-19 in tourists' destinations in China.

H2. Xenophobia is observed by Chinese from international people during COVID-19.

H3. Relationship between perceived vulnerability and ethnocentrism is observed.

#### 4.1.1. Perceived Infectability of Chinese Tourists due to COVID-19

(1) $$\begin{array}{c} \text{LPI}=f\left(\text{LCP}1+\text{LCP}2+\text{LCP}3+\text{LTX}1+\text{LTX}2+\text{LTX}3+\text{LTX}4+\text{LTX}5+\text{LTE}1+\text{LTE}2+\text{LTE}3\right)+\varepsilon , \end{array}$$

where *L* is the logarithm and PI is the perceived infectability of Chinese tourists due to COVID-19. CP1, CP2, and CP3 are bumped into or brushed against each other, destinations crowd, and feeling comfortable, respectively, which are the measurement items for crowding perception (CP). TX1, TX2, TX3, TX4, and TX5 are comfortable with foreigners, feel uneasy with foreigners, misunderstandings, suspicious, and feeling worried, respectively, which are measurement items for tourists' xenophobia (TX). Likewise, TE1, TE2, and TE3 are Chinese support the economy, everyone supports for the economy, and doing jobs, respectively, which are the measurement items for tourists' ethnocentrism (TE). *ε* is the error term.

### 4.2. Data Preprocessing

For locating data in ANN, standard techniques of normalization have not been used. For getting validation, the data preprocessing has been related to data collection. The data used A total of 823 questionnaires have been distributed in Jinan, Shandong Province, the People's Republic of China during July and August 2020 in Chinese respondents. To make the data appropriate for artificial neural networks and statistical analysis, the data have been cleaned to achieve normality. Twenty-nine respondents did not mention their age groups as per the questionnaire because they were below twenty years. The marital status was not specified by nine respondents. Similarly, thirty-one respondents from the students did not return the questionnaires. Five out of the total respondents did not mention their education level. Nineteen respondents did not disclose the number of destinations visited during the pandemic. Resultantly, 730 questionnaires out of 823 have been declared valid for ANN and statistical analysis.

### 4.3. Respondents and Method

SPSS version 21 is used for the coding and data entry process. This study focuses on the investigation of COVID-19 with the vital tourism approach. This study tests the relationship of tourism with the evolutionary tourism approach. Moreover, this study examines the crowding perception, tourists' xenophobia, ethnocentrism, and COVID-19 infection capabilities for the tourists and their influence on tourism in China. People in China are observed to be the most spenders globally on tourism, having expenditures of 277 billion USD in 2019 (UNWTO, 2019). The data are collected from Chinese tourists. A five-point Likert scale has been used to measure the perception of the local people. About 730 Chinese respondents have filled the questionnaires in different tourist destinations in Jinan, Shandong Province, and PR China. The study took place from July 1 to August 15, 2020.

The items of the questionnaire were adapted from various studies. Adaptation was compulsory to capture the most relevant data. We took the items of perceived infectability from Ackerman et al. [38], which is close to measuring the openness to coronavirus (Duncan et al., 2009). This measurement has also been established in other scopes related to diseases and influences the initiation of the behavioral immune system. The items of tourists' xenophobia were adapted from reference [60], and items of ethnocentrism were taken from reference [33]. The crowding perception items were adapted from the study of reference [30].

### 4.4. Demographic Profile

This study is performed in Jinan, Shandong Province, and the People's Republic of China. The questionnaires have been filled out by Chinese respondents. Their perception of COVID-19 and tourism has been measured. A five-point Likert scale containing measuring values of strongly disagree, disagree, neither agree nor disagree, agree and strongly agree was used to measure the tourists' perception. The respondents were divided into classes based on gender, age, marital status, tourists' mode, education, and destinations visited. Seven hundred thirty valid questionnaires were filled out by the Chinese inhabitants (Table 1). As per gender, 310 (42.46%) were male and 420 (57.54%) were female. The proportion of the female respondents is higher than males because of the visiting habits. When the data was distributed on the basis of various age groups, 160 (21.91%) were from the age range of 20–25, 235 (32.19%) were from the age range of 25–35, 180 (24.65%) were from the age range of 35–45, 90 (12.32%) were from age range 45–55, and the remaining 65 (8.90%) were from age range above 55 years. It shows most of the respondents were from the age range 25–35 years. The respondents are having an age range of more than 55 were the least.

While considering the marital status, singles were 219 (30%), married respondents were 418 (57.26%), and other respondents (widows, divorced, etc.) were about 93 (12.73%). Most of the tourists were students 395 (54.10%) and others (businesspersons and tourists) were about 335 (45.90%). As per the education level of the respondents is concerned, it was not defined for 169 (23.15%) respondents, bachelor degree holders were 234 (32.05%), master degree holders were 132 (18.08%), doctorates were 110 (15.06%), and postdocrates respondents were 85 (11.64%). The respondents were also divided based on destinations visited during and after the epidemic. About 47 (6.43%) visited only one destination, 65 (8.9%) visited two destinations, 94 (12.87%) visited three destinations, 43 (5.89%) visited four destinations, 79 (10.82) visited five destinations, and the remaining 402 (55.06%) visited more than five destinations (Figure 2).

### 4.5. Artificial Neural Network

This study is based on measuring the perception of postCOVID behavior of Chinese tourists. The brain is one of the most important organs of the human body due to direct and indirect performance. Human behavior is considered a vital source of attraction for researchers [61]. Therefore, many developmental projects have been completed due to the significant contribution of artificial intelligence [62] for solving various complex problems. For understanding the human brain, a biological neural network (BNN) has been determined to investigate the structures, functions, and features of the human brain. One of the most important consequences of these studies is the development of artificial neural networks to solve various problems.

Dendrites, somas, axons, and somas are the basic building blocks of BNN [63]. The biological structure of BNN is followed by ANN for developing some simplified mathematical model of BNN, which functions in how it works in its natural form. Similarly, reference [64] investigated that the building block of ANN is the artificial neuron. A large number of neurons are arranged in different orders to execute various tasks. The construction of various neurons provides a layered structure to ANN, composed of input, hidden, and output layers. The number of hidden layers can be increased or decreased (Figure 3).

Here, *X*_1_,…, *X*_22_ are the attributes of the respondents, including age, gender, marital status, education, tourist mode, destinations visited, bump into or brush against each other, destinations crowd, feel comfortable, comfortable with foreigners, feel uneasy with foreigners, misunderstandings, suspicious, worried, Chinese support the economy, everyone should support the economy, doing jobs, strongly dissatisfied, dissatisfied, neither satisfied nor dissatisfied, satisfied, and strongly satisfied, respectively.

### 4.6. Performance Evaluation

This study is focused on measuring the perception of Chinese tourists due to COVID-19. The performance and evaluation of the quality of services are determined by confusion matrices [65]. Various parameters are used to evaluate the performance of the predictive model. The development of a confusion matrix is considered to be one of the most vital performance evaluation matrices. A confusion matrix is a two-dimensional matrix in which rows show the actual and columns show predictive observations. True positive (TP), true negative (TN), false positive (FP), and false-negative (FN) are the basic building blocks for developing a confusion matrix (Table 2). TP shows the condition in which actual observation is positive, and the predictive model provides a positive result. TN identifies actual negative observations and positive predictive results. In the case of FP, actual observation is negative and the predictive result is positive. Likewise, in the case of FN, actual observation is positive and the predictive model result is negative. The model's performance enhances the number of TP and TN and reduces the number of FP and FN. A simple confusion matrix regarding TP, FP, FN, and TN is shown below.

Different performance evaluation parameters are calculated based on the terms listed in Table 2. The most important of these are accuracy, sensitivity, specificity, and F1 score, which are formulated as follows:

(2) $$\begin{array}{c} \text{Accuracy}=\frac{\left(\text{TP}+\text{TN}\right)}{\left(\text{TP}+\text{TN}+\text{FP}+\text{FN}\right)},\\ \text{Specificity}=\left(\frac{\text{TN}}{\text{TN}+\text{FP}}\right),\\ \text{Sensitivity or recall }=\left(\frac{\text{TP}}{\text{TP}+\text{FN}}\right),\\ \text{Precision}=\frac{\text{TP}}{\text{TP}}+\text{FP,}\\ \text{F}1\text{ Score}=\text{Harmonic mean}\left(\text{Precision, recall}\right). \end{array}$$

## 5. Results and Discussion

### 5.1. Factor Analysis

The overall Kaiser–Meyer–Olkin value is 0.82, *p* < 0.001, showing a strong validity between the constructs. High means show strong interrelationship, and low means show low interrelationship. Hence, crowding perception (CP), tourists' xenophobia (TX), and tourists' ethnocentrism (TE) are the measures to cause the perceived COVID-19 infectability (PCI). Therefore, a strong influence on the tourism sector is observed due to COVID-19 in China. High means show that tourists are in favor of the constructs. Lower means represent the disfavor of the respondents concerning a specific construct of the specific items (Figure 4). CP1, CP2, and CP3 have a factor loading of 0.76, 0.81, and 0.75, respectively. Cronbach's alpha for this indicator is 0.84 showing strong consistency. The means for these items are 4.12, 4.34, and 4.31. Also, the standard deviation for these items is 1.43, 1.54, and 1.76, respectively. TX1, TX2, TX3, TX4, and TX5 are the measurement items for tourists' xenophobia. Their respective factor loading values are 0.87, 0.74, 0.82, 0.79, and 0.81. Overall, Cronbach's alpha for this indicator is 0.83, showing strong consistency. The mean values are 3.93, 3.46, 4.17, 3.84, and 3.71. Similarly, their corresponding standard deviation values are 1.15, 1.54, 1.65, 1.44, and 1.43 (Table 3).

For tourists' ethnocentrism, TE1, TE2, and TE3 values of 0.83, 0.80, and 0.87-factor loading are obtained. Cronbach's alpha for this indicator is 0.84, showing the strongest consistency among the items. The mean values for these items are 4.09, 3.65, and 4.13. The standard deviation values of these items are 1.65, 1.85, and 1.42. Similarly, PCI1, PCI2, PCI3, PCI4, and PCI5 are the perceived infectability items having 0.81, 0.83, 0.76, 0.85, and 0.79-factor loading values. Overall, Cronbach's alpha for this indicator is 0.87 showing strong consistency. Mean values are 4.02, 4.76, 4.27, 3.96, and 3.23. Standard deviation measurements are 1.87, 1.76, 1.69, 1.87, and 1.53 (Table 4).

### 5.2. Regression

Regression analysis was conducted to measure the postCOVID perception of the tourists. As represented in the table, B values for crowding perception (CP), tourist's xenophobia (TX), and tourist's ethnocentrism (TE) are 0.367, 0.410, and 0.330, respectively, for *p* < 0.001. The results show that CP, TX, and TE directly influence perceived COVID-19 infectability (PCI) (Table 5). Moreover, CP, TX, and TE are vital factors for measuring the postCOVID-19 behavior in China. CP, TX, and TE variances are 38.20%, 30.60%, and 31.60, respectively (Figure 5).

It shows that postCOVID perception changes mostly with the crowding perception of the tourists, with an overall change of 38.20%. Tourists' ethnocentrism also influences the behavior of the tourists, prescribing 31.60% change. The least influential factor is the tourists' xenophobia of variance, prescribing 30.60% change. Hence, the results administer significant influence on the perceived infectability of COVID-19 on the tourists. Therefore H1, H2, and H3 are proved.

### 5.3. Model Training and Testing

Three subsets of the dataset have been identified for training and testing. As listed in Table 6, 70:30 ratio includes 65, 78, 91, 96, and 181 satisfaction values for high dissatisfaction, dissatisfaction (B), neither satisfaction nor satisfaction (C), satisfaction (*D*), and high satisfaction (*E*), respectively. Similarly, testing this dataset provides 36, 28, 31, 49, and 75 for A, B, C, *D*, and *E*. When the dataset is divided into a 60:40 ratio, the same satisfaction level is maintained. The output values for the training dataset are 61, 30, 95, 104, and 148 for A, B, C, *D*, and *E*, respectively. Similarly, the output values for the testing dataset are 26, 49, 37, 61, and 119 for A, B, C, *D*, and *E*, respectively.

Likewise, for a 50:50 ratio, the training output values are 29, 54, 83, 90, and 109 for satisfaction levels ranging from *A* to *E* in ascending order. Also, for testing the same dataset, we have values of 39, 67, 81, 84, and 94 for high dissatisfaction (*A*), dissatisfaction (*B*), neither satisfaction nor satisfaction (*C*), satisfaction (*D*), and high satisfaction (*E*), respectively. Resultantly, all the datasets show high satisfaction levels for most of the respondents (Figure 6).

### 5.4. ANN

ANN is used for validation in terms of data training and testing. The data are distributed into five categories: *A*, *B*, *C*, *D*, and *E*, based on the satisfaction level of the respondents for the items of the questionnaire (Table 7). The indicators of the study include crowding perception, tourists' xenophobia, and tourists' ethnocentrism. The ANN training dataset prediction values are 81, 95, 124, 143, and 167 for satisfaction levels *A*, *B*, *C*, *D*, and *E*, respectively (Figure 6).

Similarly, ANN testing dataset prediction values are 31, 49, 58, 89, and 103 for satisfaction levels *A*, *B*, *C*, *D*, and *E*. Resultantly, the respondents' high satisfaction levels regarding the items are observed (Figure 7). Hence, due to social distancing, standard operating procedures and chances of infections, due to COVID-19, have dramatically changed the life pattern of Chinese tourists in China. The changes in life patterns are observed in terms of bumping into or brushing against each other, destinations crowd, comfortable, comfortable with foreigners, uneasy feelings with foreigners, misunderstandings, suspiciousness for COVID-19, worries, support of the Chinese for the economy, support of everyone for the economy, and doing of jobs.

## 6. Conclusion

Chinese people perceived that crowding in the tourists' destinations was the root cause of spreading the virus during the pandemic. To reduce this spread, social distancing needs to be followed. Similarly, they feel uneasy, worried, and uncomfortable with the foreigners due to the fear of getting the infection in the destinations. The tourism industry in China is well-known for contributing a huge amount to the economy of the country and creating job opportunities. Hence, protective measures need to be followed to set back the industry to its original position.

In this study, an artificial neural network works as a predicting tool for measuring the satisfaction level and the perception of the tourists. For measuring the satisfaction level, the data are trained and tested for three sets of ratios: 70:30, 60:40, and 50:50. Therefore, *x*_7_, *x*_8_, *x*_9_,…, *x*_17_ show bump into or brush against each other, crowd at the destinations, comfortable feeling, comfortable feeling with foreigners, feeling uneasy with foreigners, provision of misunderstandings, suspicious visits, worried behavior, Chinese support for the economy, everyone support for the economy, and creation of jobs, respectively.

Due to cultural and social changes globally, a great influence has been observed in tourism demand. Before the epidemic, the tourism industry was the fastest growing industry in the world. This study is focused on the postCOVID behavior of tourists. A revolution has been observed in the psychology of tourists due to the spread of coronavirus in the world and the dislike of humans from other humans, and social belongingness. This research focuses on the evaluation of 730 valid questionnaires from the respondents to measure the postCOVID-19 behavior.

The results show that crowding perception, tourists' xenophobia, and ethnocentrism are the key indicators for measuring the evolutionary paradigm. The calamities have changed the psychology of the tourists. The decision continuum of the travelers has significantly changed because of the global disaster. The traveling habits of tourists all around the world have changed because of the observed mega damage.

Hence, the tourism industry is considered to be the most affected industry in the world. The findings show that crowding perception of the tourists is the most influential factor observed. Therefore, timely management of the tourist destinations is required to overcome this issue. The tourists in China need to be organized in such a manner to avoid social belongingness and reduce interaction between the national and international tourists. To avoid the adverse outcomes from tourists' xenophobia, the tourists in China need to be distributed to the national and international tourists to reduce contact between humans [66].

## 7. Implications

Insurance has become the most important issue for tourists in China. The tourists advisor companies need to bring changes in their setup to face the hard situation because of the changing global tourism environment. Standard operating procedures need to be applied in the tourists' destinations to avoid spreading the virus. Implementing such standards will ensure the health of the tourists in China. More specifically, usage of masks and gloves, social distancing, and reducing contacts need to ensure.

The usage of AI tools to predict the satisfaction level of the tourists during the pandemic is a new implication of the latest technology in the tourism sector in China. Practically, AI is applicable in customer services to involve customers and develop services in terms of convenience and flexibility. It is beneficial for incorporating tourism sectors to identify the potential factors influencing the satisfaction of the tourists.

Change orders in the tourism sector adopt crisis management policies. Free traveling in China under standard operating procedures is a vital tourism decision to be followed by the higher authorities. This is an utmost important policy for rebuilding the tourism industry. The tourism sector needs to provide confidence to the tourists. It will provide ground for the mental strength of the tourists in China. To protect against human losses, all the countries should implement protective measures to overcome the damages of COVID-19. To implement social distancing, the companies must adopt online investment systems to avoid physical involvement. To help humanity stay in the market, major companies need to adopt a no profit and no loss policy.

The role of media is of pivotal importance to come across this hard situation. The media must display such programs which can avoid depression in humans. To handle COVID-19, companies need to help the employees by giving them incentives without doing work. Complete lockdown of the markets should be implemented where COVID-19 is still spreading because nothing is more important than humanity. It is time for companies to specify corporate social responsibility funds to help the needy and poor. Irrespective of the size and complexity of the tourists' destinations, usage of masks, gloves, and sanitizers and temperature checkups must be implemented where it is difficult to lock all the business activities.

## Figures and Tables

**Figure 1:** Conceptual framework.

**Figure 2:** Graphical representation of the respondents' demographics (*X*-axis shows the attribute and *Y*-axis shows the number of respondents).

**Figure 3:** Artificial neural network showing the attributes of the data with input, hidden, and output layers.

**Figure 4:** Graphical representation of statistical values including composite reliability, mean values, standard deviation, and variance.

**Figure 5:** *R* ^2^ evaluation.

**Figure 6:** Proportional data training and testing.

**Figure 7:** Graphical representation of ANN training and testing dataset prediction.

**Table 1:** Demographic profile.

Variable (*n* = 730)	*N*	Percentage	Variable (*n* = 730)	*N*	Percentage
*Gender*			Others	335	45.90
Male	310	42.46	*Education*		
Female	420	57.54	Not defined	169	23.15
*Age*			Bachelor	234	32.05
20–25	160	21.91	Master	132	18.08
25–35	235	32.19	Doctorate	110	15.06
35–45	180	24.65	Postdoctorate	85	11.64
45–55	90	12.32	*Destinations visited*		
Above 55	65	8.90	1	47	6.43
*Marital status*			2	65	8.90
Single	219	30	3	94	12.87
Married	418	57.26	4	43	5.89
Others	93	12.73	5	79	10.82
*Tourist mode*			Above 5	402	55.06
Students	395	54.10			

**Table 2:** Confusion matrix.

	Actual observations	
Predictive model observations	TP	FP
	FN	TN

**Table 3:** Factor loading.

Constructs/items	Factor loading	Composite reliability	Mean	SD	Variance
Crowding perception (CP)		0.84			0.61
CP1. How likely are the people to bump into or brush against each other?	0.76		4.12	1.43	
CP2. Are the destinations crowded enough?	0.81		4.34	1.54	
CP3. Do you feel comfortable in the destinations?	0.75		4.31	1.76	
Tourists xenophobia (TX)		0.83			0.68
TX1. I would not feel comfortable where there are foreigners.	0.87		3.93	1.15	
TX2. I would probably feel uneasy with foreigners.	0.74		3.46	1.54	
TX3. There would be misunderstandings between foreigners and me.	0.82		4.17	1.65	
TX4. I would be suspicious towards the foreigners I encounter there.	0.79		3.84	1.44	
TX5. I would be worried that foreigners would meet me with reservations.	0.81		3.71	1.43	

**Table 4:** Factor loading.

Constructs/items	Factor loading	Composite reliability	Mean	SD	Variance
Tourists ethnocentrism (TE)		0.91			0.64
TE1. Chinese should support the economy of China by visiting during holidays.	0.83		4.09	1.65	
TE2. Everyone should support the economy by spending holidays in China.	0.80		3.65	1.85	
TE3. All Chinese should support the country by doing jobs in the tourism industry.	0.87		4.13	1.42	
Perceived COVID-19 infectability (PCI)		0.87			0.73
PCI1. If a disease like corona is around, I will get it.	0.81		4.02	1.87	
PCI2. As per my experience, if anyone around me is sick, I am likely to get sick.	0.83		4.76	1.76	
PCI3. If I got corona, I think I would have more severe symptoms.	0.76		4.27	1.69	
PCI4. I am more likely to catch infectious diseases.	0.85		3.96	1.87	
PCI5. If I get corona, it may hit me more than others.	0.79		3.23	1.53	

**Table 5:** Regression analysis.

Model	Dependent variable	Independent variables	*B*	Standard error	*t*	95% confidence interval		Hypothesis
						Lower limit	Upper limit	
	Perceived COVID-19 infectability	Crowding perception	0.367	0.052	7.057	0.231	0.416	H1
		*R* ^2^	0.382	*p* (1, 367)	46.01 *p* < 0.001			
		Tourists' xenophobia	0.410	0.063	6.507	0.145	0.362	H2
		*R* ^2^	0.306	*p* (2.123)	83.324 *p* < 0.001			
		Tourists' ethnocentrism	0.330	0.051	7.705	0.189	0.256	H3
		*R* ^2^	0.316	*p* (2.332)	51.362 *p* < 0.001			

**Table 6:** 70:30 ratio, 60:40 ratio, and 50:50 ratio for data training and testing.

70:30 ratio		60:40 ratio		50:50 ratio	
Training data set	Testing data set	Training set	Testing set	Training set	Testing set
*A* = 65	*A* = 36	*A* = 61	*A* = 26	*A* = 29	*A* = 39
*B* = 78	*B* = 28	*B* = 30	*B* = 49	*B* = 54	*B* = 67
*C* = 91	*C* = 31	*C* = 95	*C* = 37	*C* = 83	*C* = 81
*D* = 96	*D* = 49	*D* = 104	*D* = 61	*D* = 90	*D* = 84
*E* = 181	*E* = 75	*E* = 148	*E* = 119	*E* = 109	*E* = 94
Total = 511	Total = 219	Total = 438	Total = 292	Total = 365	Total = 365

**Table 7:** ANN training and testing dataset prediction.

	Predictive model observation							Predictive model observation					
Actual model observation		*A*	*B*	*C*	*D*	*E*	Actual model observation		*A*	*B*	*C*	*D*	*E*
	*A*	81	4	8	5	2		*A*	31	3	2	6	2
	*B*	5	95	4	6	9		*B*	6	49	4	7	3
	*C*	3	5	124	3	6		*C*	1	7	58	5	4
	*D*	1	7	4	143	7		*D*	4	8	6	89	8
	*E*	2	4	4	6	167		*E*	1	3	7	6	103
ANN training dataset prediction								ANN testing dataset prediction					

## Data Availability

The data collected during the data collection phase are available from the corresponding authors upon request.
